# Study of Multidimensional and High-Precision Height Model of Youth Based on Multilayer Perceptron

**DOI:** 10.1155/2022/7843455

**Published:** 2022-06-18

**Authors:** Lijian Chen, Xinben Fan, Keji Mao, Amr Tolba, Fayez Alqahtani, Ahmedin M. Ahmed

**Affiliations:** ^1^College of Computer Science and Technology, Zhejiang University of Technology, Hangzhou, China; ^2^Computer Science Department, Community College, King Saud University, Riyadh 11437, Saudi Arabia; ^3^Software Engineering Department, College of Computer and Information Sciences, King Saud University, Riyadh 12372, Saudi Arabia; ^4^Florida International University, Miami, FL, USA

## Abstract

Predicting the adult height of children accurately has great social value for the selection of outstanding athlete as well as early detection of children's growth disorders. Currently, the mainstream method used to predict adult height in China has three problems: its standards are not uniform; it is stale for current Chinese children; its accuracy is not satisfactory. This article uses the data collected by the Chinese Children and Adolescents' Physical Fitness and Growth Health Project in Zhejiang primary and secondary schools. We put forward a new multidimensional and high-precision youth growth curve prediction model, which is based on multilayer perceptron. First, this model uses multidimensional growth data of children as predictors and then utilizes multilayer perceptron to predict the children's adult height. Second, we find the Table of Height Standard Deviation of Chinese Children and fit the data of zero standard deviation to obtain the curve. This curve is regarded as Chinese children's mean growth curve. Third, we use the least-squares method and the mean curve to calculate the individual growth curve. Finally, the individual curve can be used to predict children's state height. Experimental results show that this adult height prediction model's accuracy (between 2 cm) of boys and girls reached 90.20% and 88.89% and the state height prediction accuracy reached 77.46% and 74.93%. Compared with Bayley–Pinneau, the adult height prediction is improved 19.61% for boys and 13.33% for girls. Compared with BoneXpert, the adult height prediction is improved 25.49% for boys and 6.67% for girls. Compared with the method based on the bone age growth map, the adult height prediction is improved 15.69% for boys and 24.45% for girls.

## 1. Introduction

Children and adolescents are the future and hope of the development of the country and the nation. It is a research topic of great significance to scientifically describe and predict the height growth of children and adolescents. Through the research results, experts can intervene the abnormal conditions of height growth stage in time to ensure children's normal growth.

Because of the difference in personal physical conditions and growth phase, every child has his own tempo of growth. Some of them have a high growth velocity during puberty, but this state ends early. Some adolescents have a low growth velocity, but their puberty ends late. Predicting state height during adolescents' development can determine whether the child needs medical intervention and whether the treatment for growth is effective, so as to provide the basis for clinical diagnosis [1]. Therefore, we need to find a practical model, which can accurately predict children's adult height and stage height.

The about the height growth of children and adolescents is difficult. It needs a large number of samples of normally developing adolescents. Researchers need to observe and record the multiple growth and development indicators chronically. Besides, the validation of whether the predicting adult height is correct is a long process. So, it is difficult to verify the accuracy in a short period of time. At present, statistical method is the main method in adult height prediction. It is used to classify samples and put forward prediction methods. The simplest height prediction method is the genetic height algorithm. It was proposed by Luo in Sweden in 1998, and it has been continuously improved [2]. The new genetic height prediction formula proposed in China is as follows [3]:

(1) $$\begin{array}{c} Y_{\text{boy}}=56.699+0.419*H_{\text{father}}+0.265*H_{\text{mother}}\text{,}\\ Y_{\text{girl}}=40.089+0.306*H_{\text{father}}+0.431*H_{\text{mother}}\text{.} \end{array}$$

Actually, apart from genetic factors, the growth environment also has a great influence on growth and development. So, the relative error range of genetic height and adult height is very large.

Tanner–Whitehouse method is a classical adult height prediction method [4]. It was proposed by Tanner et al. This method is based on a series of multiple regression models compiled by different sex, age, and information (menarche, height increase, and bone age increase) to predict the adult height of children. It is obvious that the calculation is too complicated. This method originated from aboard and there is a large error in Chinese children's adult height prediction [5]. Apart from that, Chinese hospitals do not have a TW3 adult height prediction model, which is adapted to Chinese children. Although some sports organizations use TW3 model, their criteria are made for the selection of athletes but not for normal adolescents' adult height prediction.

In 1952, Nancy Bayley of the University of California in the United States proposed the Bayley–Pinneau height prediction method, which is also a classical adult height prediction method [6]. In this method, the developmental types of children and adolescents are divided into early developmental type, normal developmental type, and late developmental type. This method separately calculates the three types of adolescents' proportion of heights in different bone age stages to adult height. When getting child's age, bone age, and height at present, his adult height can be determined. The prediction formula is as follows:

(2) $$\begin{array}{c} Y=\frac{H}{\text{FP}}. \end{array}$$

Here, *Y* is the predicted adult height, *H* is the current height, and *FP* is the growth rate obtained by looking up the Height Growth Percentage Table.

In addition, there is an attribute model named PB curve proposed by Preece and Baines in 1978 to describe the growth curve. In 2013, the research team also corrected three errors in the manuscript [7].

In China, the most classic adult height prediction method is the RC (radius, ulna, and short bone-Chinese wrist bone development standard) height prediction method proposed by Zhang Shaoyan using samples from five cities in Dalian, Shijiazhuang, Shanghai, Wenzhou, and Guangzhou for several years [8]. The CHN (Chinese wrist bone development standard) method of bone age assessment is performed every three months. After the bone age is fully developed, the adult height of children and adolescents is compared with the height of any bone age, and the percentile of height increase is proposed in the form of Bayley–Pinneau height prediction method. However, this method is not applicable to children in most provinces and cities in China because of the small sample size and uneven coverage.

After the millennium, many scholars have proposed new methods of predicting adult height. In 2005, Sherar et al. proposed a cumulative height velocity curve based on maturity to predict adult height [9]. In 2009, Thodberg et al. proposed an adult height prediction method based on BoneXpert automatic determination of bone age [10]. This method uses the data of adolescents from the first longitudinal study and the third longitudinal study in Zurich and the height information of parents combined with Bayesian nerves [11]. The prediction of adult height on the Internet has a very good effect. Zhang Shaoyan also conducted a study on the new Chinese bone age reference standard based on BoneXpert in 2013 [12]. In 2010, Tim J Cole combined the nonlinear mixed-effects model and proposed the SITAR (superimposition by translation and rotation) model to describe the growth trend of adolescents [13]. Based on the height and weight data of children and adolescents, Michael et al. analysed the feasibility of a series of regression models such as linear, decision tree, and random forest in predicting the direction of children's adult height. The experimental results found that the random forest regression model predicted the accuracy is better, and the adult height prediction for children aged 0–6 is better than the TW3 method based on bone age [14]. Zhi et al. screened and used 22 height-related SNP loci to construct a height prediction model from the perspective of genes. They verified it by 1220 Han populations in northern and southern China. The feasibility of the results needs further study. If more SNP loci closely related to the height of the Chinese Han population can be found, then the accuracy of the model can be further improved [15]. Shi proposed the growth trend map of children and adolescents in Zhejiang Province based on bone age. Then, he designed an algorithm based on the shortest Euclidean distance fitting to predict individual growth trends and adult height [16]. Kang established a multifeature time-series evaluation model through a neural network to evaluate the height of children and adolescents after 6, 12, 18, and 24 months of growth hormone intervention [17].

With the popularity of machine learning technology in recent years, experts and scholars in the medical field are also actively exploring the application of the multilayer perceptron model. Raoul combined floor sensors and multilayer perceptrons to interpret the sensor data to judge a person's gait pattern and predict age to determine the aging. This study is expected to have further research and applications in healthcare and medicine [3]. Boyang Su is the first attempt to predict wall shear stress in stenotic coronary arteries using multiple linear regression, multilayer perceptron, and convolutional neural network architectures in machine learning [18]. Satish selects categorical features through the AdaBoost technique and develops a new stacking technique of multilayer perceptron, support vector machine, and logistic regression. The stacking technique performs better than other models on the PIMA Indian Diabetes dataset [19]. Ertugrul uses multilayer perceptrons to predict the number of people recovering from COVID-19 to determine potential donors for convalescent (immune) plasma (CIP) treatment of COVID-19 [20]. Lee used patient information for malaria diagnosis through machine learning models. They compared the predictive performance of six machine learning models: support vector machine, random forest, multilayered perceptron, AdaBoost, gradient boosting, and CatBoost [21].

To sum up, there are difficulties in height prediction research: the long-term data are difficult to collect, the result verification cycle is long, most prediction methods are based on foreign countries' research, and the prediction accuracy rate is low. Although there are many methods for adult height forecasting, there is no unified forecasting method. With the continuous improvement of Chinese people's living standards, the previous methods are no longer suitable for contemporary children and adolescents. Through clinical diagnosis data, It was found that CHN-BP (Chinese wrist bone development standard-Bayley–Pinneau) method is generally used in Zhejiang Province to predict adult height, and the results are generally higher. The average error of prediction results for children and adolescents with developmental delays has reached 4 cm [22]. In order to accurately predict the adult height of children and adolescents, this study proposes a model based on multilayer perceptron adult height and stage height prediction for children and adolescents. The main contributions of this study are as follows:

1. Constructed adult height dataset and state height dataset. These two datasets contain children and adolescents in some cities of Zhejiang Province including Hangzhou, Shaoxing, Wenzhou, and other cities. There are 1068 data items in the adult height dataset and 45,416 data items in the state height dataset. The content of the data includes height, weight, age, bone age, and so on.
2. Adopted the optimized multi-layer perceptron model to predict adult height. In addition to age and bone age, this model added BMI to improve the prediction accuracy. The loss function was improved. So that the model training effect of height prediction can be better.
3. Compared the MLP adult height model with other models. The accuracy of boys is increased by 15.69%–25.49%, and the accuracy of girls is increased by 6.67%–24.45%.

## 2. Main Research Work

### 2.1. Datasets

Data used in this study are mainly from the students' physical health in recent years in Zhejiang Province. The number of samples with complete bone age, height, and BMI data reaches 88,752. Among the data, the student data that have been tested only once are excluded because it cannot be verified whether the model's prediction is accurate or not. Therefore, there are 11814 boys and 10894 girls with an interval of more than 1 year, and a total of 45,416 stage height data. At the same time, 1068 people's data (including 615 boys and 453 girls) were obtained from the Bone Age Research Center of Zhejiang Province, who had undergone bone age assessment and are now adults. Through telephone return visits, we obtained the adult height of these adolescents to verify if the prediction is accurate. The adult height data include gender, age, bone age, height, and weight. Tables 1 and 2 list the part of return visit data. Compared with the data collected by hospitals, the health status of the test samples taken from various primary and middle schools in Zhejiang Province is in line with the general situation. Processing the data of urban and rural schools together can better improve the generalization of the model.

### 2.2. Multilayer Perceptron

The multilayer perceptron is a mathematical model that mimics the activity mechanism of biological brain neurons. But it is not equivalent to the biological brain and nervous system. It does not rely on targets, objects, and datasets. It abstracts a certain function of biological neurons and uses simple mapping to approximate and implement complex mapping mathematical models [23].

The multilayer perceptron is promoted from perceptron. The main feature is that they have multiple neuron layers, also called deep neural networks. It is a neural network model constructed by the input layer, the hidden layer (one layer or more), and the output layer together. Compared with the single-layer perceptron, it can solve the linear inseparability problem [24].  Figure 1 shows the topology of a multilayer perceptron network with one hidden layer.

### 2.3. Adult Height Prediction

Based on the sklearn platform, this study builds an MLP regression model with adult height prediction for adolescents. The multilayer perceptron structure is designed as 3 layers: 1 input layer, 1 hidden layer, and 1 output layer. In the input layer, we select the adolescent's bone age (*x*_boneage_), age (*x*_age_), height (*x*_height_), weight (*x*_weight_), BMI (*x*_*bmi*_), and standard BMI difference (*x*_*deltbmi*_) as input values. BMI (body mass index) is a commonly used international standard to measure the degree of body weight and health. The calculation formula of the BMI index is as follows:

(3) $$\begin{array}{c} \text{BMI}=\frac{W}{H^{2}}. \end{array}$$

Here, *W* is the weight (in kilograms) and *H* is the height (in meters). Height, weight, and BMI are all important growth indicators to evaluate the growth and development of children and adolescents. Studies [25] have shown that excessive production of more aromatase in adipose tissue can induce androgen to be converted into estrogen. The estrogen represented by estradiol degrades the neoplastic matrix proteins of cartilage proliferating cells and mast cell populations. It promotes the maturation and apoptosis of cartilage mast cells, thereby accelerating the development of bone age, so that the development of obese children has the characteristics of early bone age, faster height growth, and delayed development of secondary sexual characteristics. The standard BMI used in this article comes from data released by the World Health Organization [26]. The expression formula of the input layer is as follows:

(4) $$\begin{array}{c} X_{f}=\left(x_{\text{boneage}},x_{\text{age}},x_{\text{height}},x_{\text{weight}},x_{\text{bmi}},x_{\text{deltbmi}}\right). \end{array}$$

After many experiments, the number of neurons in the hidden layer is set to 100 neurons in the male and female models [27]. In terms of the activation function, the ReLU function has a very fast calculation speed. Its convergence speed is better than the sigmoid function. It solves the disappearance of the gradient. So, we set it as an activation function. Due to the characteristics of multi-hidden-layer processing of the multilayer perceptron, it is suitable for fitting nonlinear functions. Using BP (back propagation) algorithm and by adjusting the learning rate, we can avoid falling into the local optimal solution. For the human body, height is a value that will change slightly. Measured in the morning or evening, there will be a 1 cm change in height. Therefore, in order to avoid overfitting, we do not use mean absolute error as a loss function. The expression formula of new loss function is as follows:

(5) $$\begin{array}{c} \text{loss}=\frac{1}{n}\cdot \sum_{i=1}^{N}{\left\{\max\left[0,\left(\left|d_{i}-y_{i}\right|-0.5\right)\right]\right\}}^{2}. \end{array}$$

The loss function divides the error between the expected value and the actual value into two parts: if the error is within 0.5 cm, it is regarded as the expected result; if the error exceeds the range of 0.5 cm, it is trained in a way similar to the mean square error.

The samples of male and female students with adult height data used in this article are 615 and 453. After dividing the training set and the validation set at a ratio of 3 : 1, the amount of data is limited, so all the training set data are imported in each iteration to improve the coverage of the model training samples. The result of the division of training set and test set is listed in Table 3.

After many experiments, it is finally determined that the boy's adult height network performs 46,000 iterations to achieve the optimal convergence effect. The girl's adult height network performs 48,500 iterations to achieve the optimal convergence effect. In addition, the initial learning rate is determined to be 0.00005, so that in the process of gradient descent, the network can quickly search for the optimal solution without falling into the local optimal situation.

### 2.4. Least-Squares Method

The basic idea of the least-squares method is as follows [28]: given a set of experimental data, these data are often pairs of ordinal numbers, according to the principle of minimizing the sum of squares of errors, and the best function matching of these data is found. The following is the standard formula of the least-squares method, where *P*(*x*) is the polynomial to be fitted:

(6) $$\begin{array}{c} E^{2}=\text{min}\sum {\left[P\left(xi\right)-yi\right]}^{2}. \end{array}$$

The solution process of the least-squares method is the solution process of *P*(*x*). The curve equation is set to be fitted as a polynomial of degree *n*, and the formula is as follows:

(7) $$\begin{array}{c} P\left(x\right)=a_{n}x^{n}+a_{n-1}x^{n-1}+\cdots +a_{1}x+a_{0}. \end{array}$$

The above equation is transformed into a matrix form, and the formula is transformed into *P*(*x*)=*X* · *A*, where *A* is the coefficient matrix. The formula of *X* is as follows, where *k* represents the number of points to be fitted:

(8) $$\begin{array}{c} X=\left[\begin{array}{ccccc} x_{1}^{n} & x_{1}^{n-1} & \cdots & x_{1} & 1\\ \vdots & \vdots & \ddots & \vdots & 1\\ x_{k}^{n} & x_{k}^{n-1} & \cdots & x_{k} & 1 \end{array}\right]. \end{array}$$

Both sides of the equation are multiplied by the transposed matrix of *X* at the same time to get

(9) $$\begin{array}{c} {\left(X^{T}X\right)}^{-1}X^{T}P\left(x\right)=A. \end{array}$$

Finally, the coefficient matrix *A* of the polynomial is obtained by solving the equation.

### 2.5. Average Growth Curve

According to the data in the Chinese Children and Adolescents' Height Unit Standard Deviation Numerical Table published by the Beijing Capital Academy of Pediatrics [18], the heights in the 0SD column of the male and female table are selected as the standard heights corresponding to each age, and then the least-squares method is used to fit these points. The obtained curve equation is set as the standard height curve. The average growth curve of boys and girls is shown in Figure 2.

### 2.6. Personal Growth Curve

First of all, we set the height equation obtained by the least-squares method as *H*=*f*(*x*). According to the principle of curve transformation, we add three parameters *α*, *β*, *γ*, so that the height equation becomes *H*=*f*(*αx*+*β*)+*γ*. In this formula, *α* represents the contraction and extension of the curve in the *x*-axis direction. Children with a fast puberty growth rate have an *α* value of <1, and a relatively flat child with *α* ≥ 1.

*β* represents the translation of the curve on the *x* axis. For children who develop early, the value of *β* is positive, and for children who develop late, the value of *β* is negative.

*γ* represents the amount of translation of the curve in the *y*-axis direction, and the value of *γ* in the growth curve of short children is relatively small.

The effect of the three parameters is shown in Figure 3. The solid line in the figure is assumed as the original curve *g*(*x*). Then, the dotted curve is a *g*(*αx*) curve that is compressed left and right after being affected by an *α* value greater than 1. The dashed-dotted line is the *g*(*x*+*β*) curve that is shifted to the left after being affected by the positive *β* value. The dashed line is the *g*(*x*)+*γ* curve that translates downward after being affected by the negative *γ* value.

We use the previous multilayer perceptron adult height prediction model to obtain the height as the current child's height *H*_final_ at the age of 18, and the parameter *γ* can be calculated as follows:

(10) $$\begin{array}{c} \gamma =H_{\text{final}}-f\left(18\right). \end{array}$$

Under the premise that the current age height *H*_current_ and the 18-year-old height are known, the simultaneous equations can be obtained:

(11) $$\begin{array}{c} \left\{\begin{array}{c} H_{\text{current}}=f\left(\alpha x_{\text{current}}+\beta \right)+\gamma ,\\ H_{\text{final}}=f\left(\alpha x_{\text{final}}+\beta \right)+\gamma . \end{array}\right. \end{array}$$

Due to the measurement error and the different factors of each body's constitution and growth environment, the above equations cannot accurately solve the values of *α* and *β*. The system of contradictory equations similar to the above is a problem often encountered in engineering. But, we can get a solution through the least-squares method to minimize the sum of squares of errors in each equation [29]. After obtaining the above personal growth curve, in order to verify the correctness of the curve, we substituted the age of these children in the second test into the curve equation and compared the predicted the target age height with the true value. It can be seen from Tables 4 and 5 that the prediction error is within a reasonable range, and the staged height calculated by this method is reliable. Figures 4 and 5 show the personal growth curves of the 40 children predicted by the model.

## 3. Result

After adjusting the multilayer perceptron models of male and female adolescents, the results show that the male adult height model performs well, and the maximum absolute error on the verification set is 3.25 cm. The performance of the female model is a bit worse than the male model, and its absolute error reached 5.13 cm. Due to the problem of the accuracy of the equipment and the posture of the human body during the height detection process, the obtained height data will have an error of 0.5 cm. For the human body, height is a value that will change slightly. Measured in the morning or evening, there will be a 1 cm change in height. Therefore, this study selects the difference between the predicted value and the true value within ±2 cm as the basis for accurate prediction.  Table 6 respectively lists the error and accuracy of the adult height prediction model of male and female students on the adult height verification set. This model can be used for the next stage of height prediction.

In addition, this experiment compares the adult height prediction model for teenagers based on multilayer perceptions with the traditional BP (Bayley–Pinneau) method, the Bayesian network-based BX (BoneXpert) method, and the method based on bone age growth trend map (BAGTM) to compare the prediction results of the same batch of samples. Tables 7 and 8 list a part of prediction of boy's and girl's adult height by three models. The three models' accuracy in whole test set results is listed in Tables 9 and 10.

Then, we adopt boxplots to analyse the error of this experiment. Boxplots can intuitively determine the discrete distribution of errors, understand the distribution of errors, and identify outliers in errors. The range of error is expressed by the vertical distance between the minimum and maximum values, and the interquartile range (IQR) of the error is expressed by the height of the box.  Figure 6 shows the error analysis result of boys, and Figure 7 shows the error analysis result of girls. As can be seen from Figure 6, the quartile interval and median of MLP model prediction error are better than other prediction models. As can be seen from Figure 7, the quartile interval and median of MLP model prediction error are similar to the Bayley–Pinneau method, but the number of outliers is less than the Bayley–Pinneau method, indicating that the MLP model has a better stability. Based on the above analysis, we can conclude that the performance of the MLP model prediction model is superior to other prediction models.

On the basis of the adult height prediction model, we draw the personal growth curve and predict the stage height. The experiment has a large amount of stage data for verification, which can better show the generalization of the model. Different from the above twenty-person test experiment, the data of 12,793 boys and 11,427 girls were imported into the staged height prediction model, and the corresponding next test data were used for verification. The experimental results are listed in Table 11.

## 4. Discussion

Comparing the table analysis in the experimental results, it is concluded that the multilayer perceptron model's accuracy about adult height prediction is superior to the Bayley–Pinneau prediction method and the adult height prediction method of BoneXpert, especially boys' accuracy has been greatly improved. On this basis, the individual height growth curve of each child is drawn, and then the stage height is predicted. According to the stage height prediction results in Table 6, we can put it into the growth and development diagnosis and judge whether the child's growth and development are abnormal, whether medical intervention is needed, and whether the intervention treatment is effective.

Compared with the adult height prediction model, the accuracy rate of the stage prediction model within 2 cm is about 13% lower. There are three main aspects to analyse the reasons for this situation: one is that in the process of feature learning of the MLP adult height prediction model, due to the relatively small amount of data, it cannot achieve the best results in terms of generalization. Therefore, the adult height prediction will produce certain errors. Because the data for girls in this article is relatively small, the prediction effect is worse than that of boys. The second is the error in personal curve matching. When solving equations, the least-squares method is based on the principle of minimizing the sum of the squares of the errors in each equation to obtain the values of the parameters *α* and *β*. The actual growth process of adolescents is also affected by factors such as environmental work and rest, which cannot be summarized into the model. The third is that the error of curve matching is superimposed on the error of the adult height prediction model, which expands the fluctuation range of the error, making the accuracy of the stage height lower than that of the adult height prediction.

How to solve the above situation and improve the accuracy of the model are mainly analysed in two aspects: one is to continue to adjust the neuron structure and parameters of the multilayer perceptron, increase the amount of training data, and then improve the accuracy of the adult high prediction model. The second is to optimize the method for determining the parameters *α* and *β* in the staged height prediction to improve the accuracy. The data are filtered out with an error greater than 2 cm, the characteristics are analysed, and the new methods to make state height predictions are found.

## 5. Conclusion

The adolescent adult height prediction model proposed in this study uses a multilayer perceptron to add the dimension of BMI on the basis of traditional age and bone age prediction, which improves the accuracy of adult height prediction. The experimental data of 1068 boys' and girls' adult height samples show that the accuracy rate of the boys' adult height model within 2 cm reaches 90.20%, and the accuracy rate of the girls' adult height model's prediction results within 2 cm reaches 88.89%. This model surpasses the traditional adult height prediction method. The subsequent staged height prediction model uses the least-squares method to fit the average growth curve and combines the adult height prediction results to derive a growth curve suitable for everyone. Validation of the staged height data of 12,793 boys and 11,427 girls shows that the accuracy rate of the prediction results of the stage height of boys within 2 cm reaches 77.467%, and the accuracy rate of the stage height prediction results of girls within 2 cm reaches 74.931%. Compared with the traditional height prediction method, this staged height prediction model can more intuitively show the future growth of adolescents. There are two main shortcomings of this model: there is not enough sample data with adult height and because based on adult height prediction, the accuracy of state height prediction decreases greatly. The future research work mainly has two aspects: one is to collect more samples of adult height to improve the accuracy of adult height prediction and another is to improve the prediction method of state height so that the generated growth curve is more in line with everyone's growth situation.

## Figures and Tables

**Figure 1:** Multilayer perceptron model.

**Figure 2:** Boy's mean growth curve (a) and girl's mean growth curve (b).

**Figure 3:** The influence of the three parameters of *α*, *β*, and *γ* on the function curve.

**Figure 4:** Twenty boy's individual growth curve.

**Figure 5:** Twenty girl's individual growth curve.

**Figure 6:** Male error distribution map.

**Figure 7:** Female error distribution map.

**Table 1:** Basic information of boys' return visit.

Name	Return visit date	Age (years)	Bone age (years)	Height (cm)
Wang^*∗∗*^	2018/7/26	6.00	7.08	115
Zhu^*∗∗*^	2018/7/26	7.83	8.83	125
Kong^*∗∗*^	2018/7/27	7.08	6.33	117.3
Hu^*∗∗*^	2018/7/27	8.17	6.92	123
Yao^*∗∗*^	2018/7/27	8.25	7.42	130.2
Jiang^*∗∗*^	2018/7/29	8.00	7.50	124
Xu^*∗∗*^	2018/7/29	9.83	12.83	148.4
…	…	…	…	…
Ni^*∗∗*^	2018/8/10	9.00	8.83	131
Shao^*∗∗*^	2018/8/11	10.92	12.83	148
Gui^*∗*^	2018/8/11	10.00	11.08	138.2

^*∗*^One Chinese character. ^*∗∗*^Two Chinese characters.

**Table 2:** Basic information of girls' return visit.

Name	Return visit date	Age (years)	Bone age (years)	Height (cm)
Tao*∗∗*	2018/7/21	13.6	12	155.8
Jin*∗∗*	2018/7/21	11.9	13	152.4
Zhang*∗∗*	2018/7/21	13	13.1	165
Xie*∗*	2018/7/21	11.8	12.3	150.5
Wang*∗∗*	2018/7/21	13.4	14.7	157
Hu*∗∗*	2018/7/18	11.4	11.8	148
Wang*∗∗*	2018/7/18	11.7	11.3	147
Kong*∗*	2018/7/18	11.8	11.5	144.2
…	…	…	…	…
Zhou*∗∗*	2018/8/10	11.6	11.5	142.4
Xi*∗∗*	2018/8/11	11.6	12.3	152.8

^*∗*^One Chinese character. ^*∗∗*^Two Chinese characters.

**Table 3:** The division of training set and test set unit: number of people.

Gender	Total people	Training set	Test set
Boy	615	462	153
Girl	453	338	115

**Table 4:** Twenty boys' state height prediction.

Id	Current age (years)	Current height (cm)	Target age (years)	Target height (cm)	Prediction height (cm)	Deviation (cm)
1	11.5	146.1	12.5	149.9	151.50	1.61
2	11.5	148	12.5	155.1	155.62	0.52
3	10.7	140	11.7	145	145.78	0.79
4	10.9	149.4	11.9	158.7	156.81	−1.88
5	11	148.8	12	155.2	155.32	0.12
6	11.6	151.8	12.6	157.7	158.02	0.32
7	10.9	146.5	11.9	154.8	153.93	−0.87
8	11.4	153.7	12.4	162.5	161.64	−0.86
9	11.5	146.7	12.5	154.2	153.86	−0.34
10	11.1	147.5	12.1	156.7	155.47	−1.22
11	10.6	141.1	11.6	146.6	146.90	0.31
12	10.7	144.3	11.7	151.1	151.96	0.87
13	10.8	146.9	11.8	156.5	154.43	−2.07
14	10.9	144.1	11.9	149.3	149.37	0.07
15	10.9	153.7	11.9	162.1	159.95	−2.15
16	11	150.3	12	160.2	157.89	−2.30
17	11	135.9	12	141.8	141.25	−0.55
18	11.1	157.9	12.1	164.8	166.02	1.22
19	11.3	141.7	12.3	146.7	147.33	0.63
20	11.3	138.6	12.3	147	145.01	−1.98

**Table 5:** Twenty girls' state height prediction.

Id	Current age (years)	Current height (cm)	Target age (years)	Target height (cm)	Predict height (cm)	Deviation (cm)
1	10.8	146.5	11.8	154.5	151.32	−3.17
2	11.4	146.7	12.4	154.8	151.97	−2.82
3	10.9	139.1	11.9	146.3	144.41	−1.88
4	10.7	149.1	11.7	155.7	154.31	−1.38
5	10.9	158.6	11.9	162.4	163.16	0.76
6	10.9	130.8	11.9	136.5	138.34	1.84
7	11	151.2	12	157.9	156.77	−1.12
8	11	148.4	12	155.6	153.55	−2.04
9	11	146.6	12	154.7	151.99	−2.70
10	11	149.6	12	156.3	154.80	−1.49
11	11.1	157.5	12.1	161.7	162.51	0.81
12	11.1	143.4	12.1	151.3	149.22	−2.07
13	11.2	153.2	12.2	158.1	158.44	0.34
14	11.2	156.8	12.2	160.5	160.49	−0.01
15	11.5	165.4	12.5	168.3	169.89	1.59
16	11.6	139.9	12.6	148.6	145.16	−3.43
17	11.7	158.4	12.7	161.4	161.38	−0.01
18	11.5	146.4	12.5	149.9	151.96	2.06
19	10.9	150.4	11.9	159.4	155.75	−3.64
20	10.8	141.1	11.8	149	147.11	−1.88

**Table 6:** Result of adult height prediction model.

Comparison of model results	Boy	Girl
Mean absolute error (cm)	1.04	1.08
Root mean square error	1.28	1.60
Mean absolute error in 2 cm	90.20%	88.89%
Mean absolute error in 1 cm	60.8%	60.00%
Absolute value of maximum error (cm)	3.25	5.13

**Table 7:** Male generation year height prediction results table.

Age (years)	Bone age (years)	Weight (kg)	Height (cm)	Adult height (cm)	Predict adult height (cm)			
					BP	BX	BAGTM	MLP
6.0	7.1	18	115	170.5	170.1	167.0	169.1	167.2
7.8	8.8	26.5	125	168	173.6	166.0	169.4	169.6
7.1	6.3	24	117.3	171	168.8	164.3	173.4	170.3
8.2	6.9	21	123	172	171.3	165.2	176.4	171.2
8.3	7.4	27	130.2	180	183.6	171.8	183.0	178.7
8.0	7.5	23	124	174.8	174.9	165.9	174.3	172.1
9.8	12.8	53	148.4	174.6	174.6	172.0	172.3	174.4
9.0	8.8	23.5	131	174.2	174.2	169.0	173.6	173.6
10.9	12.8	44.5	148	175	174.1	169.6	171.9	172.8
10.0	11.1	39	138.2	173.5	178.1	170.3	171.2	171.8
10.5	10.5	30	136.6	171.8	171.8	167.4	172.2	172.2
10.9	11.1	26	134	166.5	165.0	163.1	167.7	166.4
11.8	12.8	31	144.7	169	170.2	166.3	169.7	167.3
11.2	12.8	54	154	178	181.2	175.8	175.4	176.9
11.7	13.2	51	163	183.5	188.9	181.7	179.7	184.7
11.9	12.7	36	141	165	163.4	163.8	166.6	166.4
11.3	11.5	34	141	172.5	172.4	168.6	172.2	171.7
12.3	12.6	44	152.2	176	176.4	173.9	175.1	176.8
12.0	13.2	33.5	148	170	171.5	166.9	169.6	168.6
12.6	13.1	46	148.5	168	166.9	166.4	170.1	169.6
13.6	14.5	43	156.5	166.5	165.1	165.4	167.8	166.5
13.2	13.0	32.5	151.3	170	172.7	169.4	173.3	170.6
13.1	13.5	39	158	174	175.2	173.1	173.7	174.2
14.2	15.2	50	163.5	169	169.1	168.7	169.7	168.7
14.8	16.0	52.5	165	168.5	168.4	168.2	167.2	167.9
14.5	15.2	65	164.5	170.5	169.1	169.4	169.3	169.8
15.0	15.8	77	165	169	168.0	168.6	167.9	168.2
15.4	17.5	95	165.3	165.3	165.3	166.8	165.6	165.8
15.4	17.0	63	162.5	163.5	164.1	164.4	163.0	163.3

**Table 8:** Female generation year height prediction results table.

Age (years)	Bone age (years)	Weight (kg)	Height (cm)	Adult height (cm)	Predict adult height (cm)			
					BP	BX	BAGTM	MLP
9.5	10.2	20	125	146	143.0	148.7	149.0	146.1
11.1	11.0	29	133.7	147	147.6	150.9	152.5	150.0
10.9	12.2	33.5	136.7	149	149.7	150	148.3	149.1
12.2	12.8	42	145.3	150.5	151.7	153.5	153.8	155.3
6.8	7.3	20	114.5	151	148.3	151.5	153.6	153.7
6.1	5.1	16	105.4	152.8	143.8	150.7	155.1	152.3
9.6	9.6	22	128.5	153	150.6	151.1	155.1	153.3
7.5	8.8	20.5	120.6	153.8	152.7	153	153.0	153.0
8.5	11.2	35	136	154	153.3	157.7	153.5	152.6
7.5	9.0	21	121.3	154	153.5	153.2	152.6	153.5
9.9	11.5	40.5	138.5	154.5	155.4	155.4	154.2	153.8
9.9	9.7	23	130.2	156	152.6	154.3	155.8	154.2
5.3	6.0	18	111.3	156	154.6	157.3	155.1	157.6
7.0	7.4	23	118.8	156	153.9	155.6	156.8	156.8
9.9	11.5	37.5	139	156.5	156.0	156.5	154.7	154.5
13.8	14.7	40	155.3	157.5	157.2	157.7	157.3	157.4
11.7	11.8	31	146.5	158.2	158.9	158.2	159.1	160.0
10.0	11.2	51	142.3	158.5	160.4	160	158.4	158.1
11.9	13.0	38.5	152.4	159	161.3	159.9	159.2	161.0
11.8	12.3	36	150.5	159.5	159.9	159.3	160.9	161.3
13.4	14.7	52	157	159.5	159.7	159.9	159.0	159.5
9.4	11.7	39	143.2	159.6	159.6	161.4	156.4	158.3
9.8	12.2	37.5	147.3	159.8	161.3	161.1	157.8	159.8
10.5	11.5	29.5	144.4	160.2	162.1	159.8	157.3	160.4
10.2	8.0	24	133.5	166	166.0	159.1	172.0	165.1
12.2	12.0	47.5	154	167	167.0	163.5	165.6	166.1
13.6	12.0	38	155.8	167.2	167.2	163.3	167.4	168.6
12.4	12.0	36	148	160.5	160.5	159	160.1	160.4
13.0	13.2	44	165	172	170.6	170.8	171.4	172.1

**Table 9:** Comparison of boy's adult height prediction.

Model	Accuracy (%)	Mean absolute error(cm)	Root mean square error
MLP	90.20	1.04	1.28
Bayley–Pinneau	70.59	2.10	3.07
BoneXpert	64.71	2.55	3.39
BAGTM	74.51	1.44	1.10

**Table 10:** Comparison of girl's adult height prediction.

Model	Accuracy (%)	Mean absolute error (cm)	Root mean square error
MLP	88.89	1.08	1.60
Bayley–Pinneau	75.56	1.38	2.09
BoneXpert	82.22	1.60	2.07
BAGTM	64.44	2.02	1.68

**Table 11:** Comparison of boys' and girls' state height predictions.

Comparison of results	Boys (12793)		Girls (11427)	
Deviation	Amount	%	Amount	%
Within 1 cm	5428	45.945	4809	44.143
Within 2 cm	9152	77.467	8163	74.931
Within 3 cm	10949	92.678	9955	91.381
Mean absolute error	1.3497		1.4054	

## Data Availability

The dataset used to support the findings of this study was supplied by the Zhejiang Provincial Bone Age Research Center in China, under license, and the dataset involving privacy cannot be shared.
